# The Role of Community Participation in Planning and Executing Malaria Interventions: Experience from Implementation of Biolarviciding for Malaria Vector Control in Southern Tanzania

**DOI:** 10.1155/2022/8046496

**Published:** 2022-09-23

**Authors:** Athuman Yusuph Matindo, Albino Kalolo, James Tumaini Kengia, Ntuli Angyelile Kapologwe, David Zadock Munisi

**Affiliations:** ^1^Department of Health, Musoma District Council, Mara Region, Tanzania; ^2^Department of Public Health and Community Nursing, School of Nursing and Public Health, The University of Dodoma, Tanzania; ^3^Department of Public Health, St. Francis University College of Health and Allied Sciences, Ifakara, Tanzania; ^4^Center for Reforms, Innovation, Health Policies and Implementation Research (CeRIHI), P.O. Box 749, Morogoro Road, Makole (Near Bunge Premises) P.O. Box 749, Dodoma, Tanzania; ^5^Department of Health, Social Welfare and Nutrition Services, President's Office Regional Administration and Local Government (PORALG), Dodoma, Tanzania; ^6^Department of Microbiology and Parasitology, School of Medicine and Dentistry, The University of Dodoma, Tanzania

## Abstract

**Background:**

Malaria remains a disease of great public health importance in 85 countries globally. Developing countries face resource constraints in implementing public health interventions aiming at controlling malaria. Promoting community participation may contribute to rational and effective use of resources and therefore facilitating achievement of intervention goals in a cost-effective manner while fostering sustainability. However, this can be possible if the community is engaged at all stages of the intervention, from designing, implementation, monitoring, and evaluation of results. This study aimed at understanding community participation in the implementation of a biolarviciding intervention for malaria vectors control in Southern Tanzania.

**Methods:**

The current study adopted explanatory mixed method study design in collecting data. Quantitative data were collected from 400 community members and 12 vector control coordinators using structured questionnaire while qualitative data was collected through key informant interviews to 32 participants and in-depth interviews to 5 vector control coordinators who were purposively selected from the 12 councils. Quantitative data analysis involved descriptive and inferential statistics. Thematic analysis was used to analyse qualitative data.

**Results:**

Of 400 community members, only 90 (22.5%) participated in biolarviciding implementation. Predictors of community participation were willingness to participate (AOR = 3.15, 95%CI = 1.14 − 8.71, *P* value = 0.027) and community involvement (AOR = 6.07, 95%CI = 2.69 − 13.71, *P* value < 0.001). The study revealed that the main barriers to community participation were lack of effective involvement and lack of incentive to community volunteers while high willingness to participate was a facilitating factor for community participation.

**Conclusion:**

The study revealed low community participation in biolarviciding implementation in Southern Tanzania with willingness to participate and community involvement being the main predictors for community participation while lack of incentive to community volunteers was one major barrier to community participation. This explains the persistence of an unresolved challenge of community participation in malaria interventions. Therefore, more efforts are needed to improve the participation of community members in Malaria interventions through advocacy, awareness creation of respective roles, and responsibilities of the community members and fostering community ownership. Additionally, councils need to design customized motivation package for the community members.

## 1. Introduction

Malaria remains a disease of great public health importance in 85 countries globally [1, 2]. The World Health Organization (WHO) African region carries the highest burden [2, 3]. In the year 2020, it was estimated that about 7.2 million malaria cases occurred in Tanzania [4]. Existing efforts to control malaria include the use insecticide-treated mosquito bed nets, application of indoor residual spray, and increased access to early detection and treatment with artemisinin-based combination therapy [5, 6]. To complement the existing efforts toward malaria control and elimination, in the year 2017, Tanzania scaled up a nationwide biolarviciding program for mosquito control in both urban and rural areas [7, 8]. The intervention has the following benefits; assist in fighting against mosquito resistance to insecticides reported in the country; reduce outdoor biting mosquitoes, thus preventing outdoor malaria transmission; and assist in control of other mosquito-borne diseases transmitted by mosquito such as Culex and Aedes species [9–12]. In Tanzania, the implementation of biolarviciding is done by councils through their health department and in collaboration with community members, and it involves breeding site identification and application of biolarvicide to identified waterbodies and surveillance.

Scaling up of public health intervention in resource limited countries like Tanzania is likely to be challenged by financial and human capital constraints [13–15]. Innovative ways that promote community participation provide promise toward effective and efficient implementation of these interventions since through community participation people can volunteer in activities or donate equipment, fund, and other resources involved in the implementation [16]. Community participation is a process through which community influence and share control over development initiatives and the decisions and resources which affect them [17]. Community participation comprises of two terms; community involvement this entails making the community aware of all the steps involved in the project, and community engagement which is the actual involvement of the community in the execution of project activities. It is determined through engagement of community members in four components of intervention; engagement in needs assessment, resource mobilization, community organization, and program management [17].

Community needs to participate in identifying the problem of their priority and planning for solution to solve them [18]. Community members should also be willing to contribute the resources required for implementation which can be in terms of time, labour, fund, or material required [19]. In order to effectively take part in implementation, they need to be integrated through groups that are tasked with a specific role and well-coordinated. This organization ensures smooth running of activities and enhance community cohesion among members and a positive attitude toward the intervention [17, 20]. It is therefore important to fully involve the community members in the whole process of biolarviciding for effective implementation and sustainability of the intervention while promoting the culture of the said practice.

Community involvement requires that community members are fully involved at all stages especially at the designing and planning phase which enhance the acceptability of intervention among the community members and foster community engagement [16, 20]. Involving community members at various stages of implementation helps to influence and share control over development initiatives, which enhance a sense of community ownership and influence community support in generating resources, contribution of ideas, and leadership during program design and implementation [16, 21]. Such benefit has been evidenced through case studies conducted in Tanzania and elsewhere in the world [20, 21]. In this way, community involvement facilitates successful implementation of the intervention in a cost-effective manner while raising community pride and cohesion, which are essential factors for the success and sustainability of interventions [21]. A program that requires community participation like biolarviciding, if designed and directed by government officials without community involvement, may fail or lack sustainability when implementing partners or government withdraws support [16, 22].

The implementation of biolarviciding in Tanzania was meant to be community-based and led, in which community participation is vital for its success [10]. According to national guideline on biolarviciding, community need to take part in designing and planning for implementation and take part in activities such as breeding site identification and biolarvicide application in their respective areas. However, attainment of effective community participation is a complex process, since the community is a heterogeneous entity, consisting of people with different social status and behaviour, thus differ in their abilities and interests toward participation in community activities [23]. This complexity of community participation together with the past experience on implementation of the malaria interventions in Tanzania which pointed to less involvement of the community in both planning and implementation inspired our team to conduct a study to understand the community participation in the biolarviciding intervention for malaria vector control in Southern Tanzania [24, 25].

## 2. Material and Methods

### 2.1. Study Site

The study was conducted in Lindi and Mtwara regions in the Southern Zone of Tanzania. The two regions are among 26 regions of Tanzania mainland. Administratively, the southern regions have been divided into 15 councils as follows: six councils for Lindi region; Liwale District Council, Kilwa DC, Lindi DC, Nachingwea DC, Ruangwa DC, and Lindi Municipal Council; and nine councils for Mtwara region; Mtwara MC, Mtwara DC, Newala DC, Newala TC, Tandahimba DC, Masasi DC, Masasi Town Council, Nanyamba Tc, and Nanyumbu DC [26]. These regions have relatively high prevalence of malaria as reported in the Tanzania Malaria Indicator Survey (TMIS) of 2017 [3] where the prevalence of malaria in under-five age children was 12% for Lindi and 15% for Mtwara. According to 2012 population census projections, the zone is home to over 2,135,506 people with 864,652 being in Lindi region and 1,270,854 being in Mtwara region [26].

### 2.2. Study Design and Approach

The present study adopted explanatory mixed method study design in which quantitative data were collected and analysed then followed by qualitative data. The quantitative component is aimed at collecting information related to the extent of community participation and their determinants. The qualitative component is aimed at gaining an in depth understanding on experience and other contextual issues surrounding community participation. This design helps “to obtain different but complementary data on the same topic” to best understand the research problem [27].

### 2.3. Sample Sizes and Sampling Procedures

A total of 15 vector control coordinators (VCC), one from each council, were expected to participate in the study; however, only 12 participated. Sample size for community members was computed using the Kish and Leslie formula [28].

In the calculations, we used community participation of 50%. The level of significance was set at 95% and level of precision at 5%. Adding 5% nonresponse rate, a total sample size of 404, we managed to recruit a total of 400 community members. Then from each region, two councils were selected, one (1) urban council, i.e., municipal council and one (1) rural council, i.e., district council. Because each region has one urban council (municipal council), this was conveniently sampled, then, from the remaining rural councils, one was randomly selected; then, 100 community members were selected from each of the four councils. The study involved only community members who were aged above 18 years, able to provide consent and who were residents in the area for not less than a year. Vector control coordinators were conveniently selected while community members were selected through stratified sampling.

### 2.4. Data Collection Tools and Methods

#### 2.4.1. Quantitative Data Collection

Data were collected using structured questionnaires. The questionnaires were administered by the researchers and trained research assistants to community members while self-administered to vector control officer. All questionnaires were prepared in English. Questionnaires for interviewing community members were then translated into Kiswahili.

The questionnaires captured information on sociodemographic characteristics, community awareness on biolarviciding, community involvement, willingness to participate which were treated as independent variables, and community participation as dependent variable. Willingness to participate was obtained through interviewing the community members on four components; preference to provide opinion, preference to take part in activities, and likelihood to find time and contribute resources. To understand the community participation, community members and vector control coordinators were interviewed separately based on relevance of the group in the implementation process. Community members were interviewed on their participation in need assessment, activity engagement (breeding sites identification and biolarvicide application exercise), and engagement in program management, while vector control coordinators were interviewed using modified spider gram model of participation through focusing in four areas: involvement in planning, organization, volunteer for activity, and program management [17]. Each component carried 1 mark. Total score was 0 to 4. The level of community participation was then graded in accordance to the model with minor modification, as there were 400 community members, an average score with value of 0-2 was regarded as low, and an average score of 3-4 was regarded as high.

#### 2.4.2. Qualitative Data Collection

Qualitative data were collected through key informant interview (KII) of community leaders, village chairpersons and members of village health committee, and in-depth interview (II) to vector control coordinators. This sought to understand the extent of biolarviciding implementation and likely barriers stemming from resource availability, community involvement, community willingness to participate, and community participation: involvement in the needs assessment and their actual engagement through community organization, contribution of resources, identification of the breeding sites, biolarvicide application, and program management in respective villages or streets. Interview guides, notebooks, and audio recorder were used for guidance and gathering interview information. The interview guides were prepared in English and translated into Swahili for ease communication. The tool was adopted (modified) from the recommended tool for conducting scaling up case studies developed by WHO in collaboration with Expand Net and Management System International staffs of 2007 [29] and used in the study done by Quintero et al. in 2017 [30].

### 2.5. Data Management and Analysis

#### 2.5.1. Quantitative Data Processing and Analysis

Data were entered into SPPS version 20 for management and analysis. Age was grouped into 15-24, 25-54, 55-64, and above 65 based on labour working group classification [31]. Stratification of occupation and education level was based on existing reports on socioeconomic profiles [32, 33]. Proportion of community members according to age group, council of residency, awareness, involvement, willingness to participate in biolarviciding (as independent variables), and participation in either of biolarviciding activities (as dependent variable) was computed. Then, determination of association between independent variables and dependent variable was done by using logistic regression, beginning with univariable logistic regression followed by multivariable logistic regression analysis.

#### 2.5.2. Qualitative Data Processing and Analysis

Data processing and analysis was guided by framework of analysis as described by Gale et al. [34], whereby data from both key informants and in-depth interviews were transcribed by researchers who conducted the sessions, then translated into English by a Linguist. The transcribed and translated information were then entered into “ATLAS.ti” version 8 for data management and analysis. Thematic analysis was performed whereby the transcription verbatim was interpreted into codes that were generated inductively by three interdependent coders, latter grouped into categories which were merged to generate themes.

### 2.6. Integration of Findings

Findings from qualitative and quantitative data were integrated after completion of data analysis using a triangulation approach [27], whereby interpretation of quantitative data was followed by qualitative to provide complementary information that appeared to converge or contradict one another. This helped to provide comprehensive information on objectives under study.

## 3. Results

### 3.1. Sociodemographic Characteristics of Community Respondents

A total of 400 community members were recruited in the study. The age of participants ranged from 18 to 82 years with a mean of 41 (15.37SD). It was observed that most of the participants were aged 25-54 (69.3%), married (52.8%), farmers (62.3%), and had primary education (55.3%) (Table 1).

### 3.2. The Level of Community Participation in Biolarviciding Implementation

Out of 400 community members, only 13 (3.25%) study participants admitted participating in some biolarviciding implementation activities such as detection of breeding sites and application of biolarvicide, 5 (1.25%) contributed equipment, and 15 (13.25%) assisted in program management. Overall, majority 339 (84.75%) of community members did not participate in biolarviciding implementation while only 61 (15.25%) reported to participate (Figure 1).

There was a difference in the level of community participation across demographic characteristics. Residents of Lindi municipal council 29 (29%) showed higher participation than residents from the rest of the councils. It was further noted that highest participation was among respondents of 55 to 64 age group 9 (23.1%), while participation was almost similar with males having participation rate of 29 (14.6%) and female, 32 (14.9%). Married respondents 39 (18.0%) had higher participation rate as compared to unmarried participants 22 (11.1%). Participants with primary education and with formal employment had higher participation rate 40 (18.6%) and 5 (19.2%) than other groups, respectively (Table 2). Analysis using modified spider gram model indicated an average value of less than 1 (0.3175) which indicates low community participation (Table 3).

We further asked the vector control coordinators on the extent to which community members were engaged in biolarviciding implementation. Of 12 vector control coordinators interviewed, 10 (83.33%) suggested low level of community participation. Further item analysis showed 6 (50.0%) of them had involved community leaders in the need assessment for biolarviciding implementation, 7 (58.33%) reported poor organization among staff involved in biolarviciding, and 2 (16.67%) reported to have been assisted by community leaders in mobilizing community members to volunteer for activities and equipment donation while only 1 (8.33%) vector control coordinator reported leaders were involved in the biolarviciding program management (Table 4).

Similar findings were obtained from qualitative data where only a few of interviewees showed to have participated in biolarviciding implementation.

*Some people are understanding [participating] while others do not (KI 7, Female, Community leader).*

Despite reporting low community participation, both sides; community leaders and vector control coordinators acknowledged the participation of community members in various activities; from identification of breeding sites to application.

*As a chairperson, I have to show them all the areas with standing water. I showed them all water that runs from toilets and all areas with standing water (KI 7, Female, Community leader).*

*The community members collaborate with us by showing the areas with mosquitoes' breeding that we do not know. They tell us when there is a place we forget (IDI 2, Male, Vector Control Coordinator).*

Some of interviewees reported that those who participated required payment, without which they could not continue with activities, and therefore, it was necessary to allocate fund for paying them. However most councils could not afford to set aside fund as incentives to those taking part in biolarviciding activities.

*We pay them. As I told you we requested fund for this activity. Unfortunately, the fund was not all released. So, the amount that was endorsed, we hired spraying machine, and the rest amount we paid these labours. We paid them 30,000 (almost 13 USD) each (IDI 5, Male, Vector Control Coordinator).*

*The group has been very helpful in facilitating this activity. However, they started as volunteers in the beginning but, in the end, they started demanding for allowances. Since the district council could not pay them, their participation decreased (IDI 1, Male, Vector Control Coordinator).*

### 3.3. Level of Community Awareness and Involvement on Biolarviciding Implementation

Of the 400 respondents, 49 (12.25%) were aware of biolarviciding implementation while 351 (87.75%) were not aware of biolarviciding implementation in their areas. It was further observed that out of the 400 interviewed community members, 49 (12.250%) were involved in planning for biolarviciding implementation while 351 (87.75%) were not involved.

Consistent with survey results, interviewees reported low involvement of leaders in biolarviciding. Only a few reported to have been involved during planning while majority were not involved at any stage.

*Usually, we do not get involved when things are planned in this council, only that when they come for the exercise (KI 7, Female, Community leader).*

*We have never been consulted but we heard that some people move around our areas to apply biolarvicide in those areas with standing water. However, we do not know anything about it because they never told us that they would come to our area on a certain day (KI 2, Male, Community leader).*

It was noted that some of the interviewees were not aware of the implementation, and they suggested that it was important to involve the community for program sustainability.

*If they applied without informing us, I beg them in next round they should involve us so that we can understand what they do, so that we can sustain it (KI 35, Male, Community leader).*

When probed as to why some of the community leaders were not involved in the activity, and some vector control coordinators responded that the leaders were not always available in the meetings or during the activity. It was also reported that it was sometimes difficult reaching all villages for meeting leaders, especially those leaving in remote areas due to lack of reliable transport.

*We normally attend full council meeting where ward leaders are members and as representatives of village leaders. So, all directives that we want to communicate to villages community members, we deliver them to the District Medical Officer, who also attends full council meeting, and we believe the messages get to the village leaders (IDI 5, Male, Vector Control Coordinator).*

*I went to some places to inform them about the activity, but I was unable to reach those in very remote areas (IDI 9, Male, Vector Control Coordinator).*

*Because of different life challenges, some of the street/village leaders are not found in their places at the time when the Heath Officer get to their places (IDI 2, Male, Vector Control Coordinator).*

### 3.4. Level of Willingness to Participate in Biolarviciding Implementation

Of 400 respondents, 352 (88.0%) showed willingness to provide opinion for biolarviciding, 334 (83.50%) showed willingness to take part in biolarviciding activities, 304 (76.0%) were likely to find time to take part in biolarviciding, and 282 (70.50%) showed willingness to contribute fund. The mean contribution amount per household per year was TZS.1,855 (almost 0.8 USD). Overall, 311 (77.75%) showed high willingness to participate in biolarviciding implementation (Table 5).

All interviewees agreed that it is important to apply biolarvicide in mosquito breeding sites and that themselves and the community members would be willing to participate in future implementation.

*Since we have been the victims of Malaria, I think the community would be willing to participate in destroying the mosquito breeding sites without asking for payment (KI 10, Male, Community leader).*

Although there was high willingness to participate in the activity, it was not likely that community members would keep volunteering for a long time. One interviewee reported that those volunteering for the activity would need to be paid some amount.

*They would be willing to participate but under normal circumstances, they would require payment despite the benefit they get as a result of the activity (KI 29, Female, Community member).*

*Nowadays things have changed, especially among youths. Most of them are educated, but all they want is payment. You can train them but once they have received such knowledge, they take it as an asset, a tool to earn money (KI 31, Male, Community member).*

Interviewees reported the community would be willing to contribute if they were encouraged to contribute a reasonable amount of money. Majority proposed the amount between TZS.500 (almost 0.2 USD) to 1000 (almost 0.4 USD) per month of application.

*That could be possible. What I am saying is that they need to inform us the leaders, they need to encourage us! That could be possible! We do contribute some money for cleanliness, we do contribute regardless of our financial challenges. We could afford it at our capacity (KI 8, Male, Community leader).*

*Maybe 1000 per every family when they come to apply biolarvicide. People will understand [accept to contribute] (KI 7, Female, Community leader).*

However, some community leaders expressed concerns regarding proposing contributions from community members. They suggested the difficulty could be due to financial incapability.

*They will positively receive it. But as life has become difficult these days, it is not a good idea to ask people to contribute some money. I cannot speak for them but I see it difficult to implement (KI 4, Female, Community leader).*

*Yes [they might contribute]. But it depends. Because some people would think this is the role of government or may be officials have abused allocated fund for this activity and in turn they want contributions as a replacement. But with sensitization it is possible (KI 23, Male, Community leader).*

### 3.5. Univariable and Multivariable Logistic Regression Analysis for Factors Associated with the Level of Community Participation in Biolarviciding

Univariable and multivariable logistic regression analysis for factors associated with the level of community participation on biolarviciding was performed. Results indicated that the odd of participating among those with high willingness to participate was 3 times higher than the odd of participating in those with low willingness to participate (*P* value = 0.027), while the odd of participating among those who were involved was 6 times higher the odd of participating in those who were not involved (*P* value < 0.001) (Table 6).

The benefit of awareness creation and involving the community members in enhancing community participation was also reported by some of interviewees. Information from interview suggested that if they are involved, they can support doing activities involved in biolarviciding.

*Just like I said, we consulted sub-village leaders and they helped us in finding the youths to work with and in the end, the activity was done. [That means] people understand it, they agreed to work with us (IDI 3, Female, Vector Control Coordinator).*

*My community would participate; what is important is to encourage them because it is an activity that is important for them. If I encourage my people, I believe that they would participate (KI 2, Male, Community leader).*

*That could be possible. What I am saying is that they need to inform us the leaders, they need to encourage us! That could be possible! (KI 8, Community leader).*

Likewise, the willingness among the community members enhanced their participation in biolarviciding. One reported some community members having high willingness which made the application successful.

*They showed to be willing to participate. They had a great contribution in the activity. We would have not succeeded without their support. There was a need to use some equipment. The exercise was difficult, there were no boots, no masks but people did it voluntarily (IDI 3, Female, Vector Control Coordinator).*

## 4. Discussion

It has been reported that community engagement is central for long-term success and sustainability of any community based intervention [35]. Studies have further reported that interventions in which community members had been fully involved tend to be cost-effective and sustainable [16, 22]. Recently, practitioners, policymakers, and researchers have been engaging community members in public health interventions [21], as such, efforts to scale up biolarviciding for malaria vector control would require an understanding of the current level of community participation. This study assessed the level of community participation in biolarviciding for malaria vector control in the study area therefore contribute to the few available literature on community participation in malaria interventions in Tanzania.

The study found low community participation as perceived by all the participants. This was determined through assessing the engagement of community members in four main areas as described by Chilaka [17]; needs assessment, organization, resource mobilization, and program management. Need assessment involves engaging the community in identifying the priority health problem and developing mutual goals and strategies toward addressing it [36]. This helps the community take part in developing an inclusive action plan for addressing the identified problem and in turn increases their participation in implementation and evaluation of a relevant intervention [37]. It was observed that more than half of community members and their leaders did not take part in needs assessment for implementation. Developing individual and community engagement through this “bottom-up” approach to participation is known to create a positive behaviour change though it requires development of a strong interactive community infrastructures [38, 39]. Lack of full engagement of community in need assessment affects the organization and engagement in implementation of the developed action plan [17].

Community organization ensures that each group of the community members is tasked with a specific role and are well-coordinated. This organization ensures the smooth running of activities and enhances community cohesion among the members and a positive attitude toward the intervention [17, 20]. A well-coordinated system facilitates quick decision and implementation of the intervention [17]. This study observed no clear assignment of task and good coordination between the expert and the community. This reduces a sense of program ownership, thus discourages the community from participating fully as manifested in this study where less than a quarter of community members were engaged in any of the activities for biolarviciding. Similar observation was noted among community leaders where more than two thirds did not engage in any activity.

Major factor affecting community participation among councils was low involvement of community members in implementation process. Community involvement fosters community participation and sustainability of intervention [16, 20, 22]. According to the guidelines governing biolarviciding, community need to be made aware of the implementation right from the beginning in order for them to know what precautions need to be taken when biolarviciding operations are going on and thereafter [40]. Similarly, community members had to get involved in various stages of implementation; planning and execution of activities involved in biolarviciding [10]. It was found that less than a quarter of community members and only of half community leaders were aware of biolarviciding implementation. On the other hand, more than two thirds of community members and community leaders had been consulted at either stage of implementation. These results are similar to the findings in the study done at Iringa region, Southern Highlands of Tanzania [25]. In this study, it was noted that there was significant variation in participation rate across councils, with Lindi Dc reporting the highest participation rate. Several factors have been reported to facilitate community participation, and one such factor is community leadership which has been reported to vary across communities [41]. In this case, there are likely community leadership differences across different councils that might have led to the observed differences in community participation. To enhance our understanding on community participation, any underlying differences between councils that might influence community participation should be explored. Studies has further indicated that one of the most common reported barriers to participation is being too busy, and this seems to be less important as one ages. This study noted that participants of the age between 55 and 64 years had higher participation than other age groups. This could be because of the fact that participants in this age group are typically less busy as compared to the youth [42].

Despite low community participation, community members expressed high willingness (77.75%) to participate in biolarviciding, both in engaging in activities and contributing resources to support the implementation. The finding of this study was as nearly similar to findings reported in as study done by Mboera et al. [43] which reported respondent willingness to pay at 73.1%. However, the affordable amount proposed by respondents per household per year was Tshs.1855/=, which was equivalent to US$0.80 [44], quite below the estimated cost for biolarviciding requirement as shared by Rahman et al. [45] that estimated a household payment of US$ 6.18 per household per year. This highlights unreliability of community members in donating sufficiency fund for implementation, thus, the government needs to play a great role in availing fund for biolarviciding implementation.

Finally, the study revealed lack of motivation among the community volunteer as the contributing factor to low community participation. It was reported by vector control coordinators that some of the community volunteers could not maintain their participation due to lack of incentives. Likewise, some community members shared that “*things has changed*,” and the current community especially young population requires some incentive to maintain their engagement. Some councils did not allocate fund for motivating those who take part in activities, expecting them to work without payment. As a result, in the long run, the volunteers could not continue with taking part in activities. Similar findings were found in the study done in Dar es Salaam, Tanzania [46]. Unless this important factor taken into consideration, it will be unlikely to sustain community participation in biolarviciding for malaria vector control.

## 5. Conclusions and Recommendations

In conclusion, the study showed low community participation in biolarviciding implementation among community members in councils of Southern Tanzania. Low community involvement and lack of motivation to community volunteers were identified as major factors that affect community participation.

Implementers should promote community participation through advocacy and community sensitization to create awareness and later involvement in all stages of biolarviciding; from planning, execution, and evaluation of the implementation activities. This will help in reducing resource gaps through contributing resources and volunteering for the activity. Also, it is important for councils to allocate fund in order to provide incentives to those involved in biolarviciding that will attract sustainable participation in the implementation.

## 6. Strength and Limitations

The study has strength in that it employed mixed method, quantitative and qualitative approach, and triangulation of study population which ensured rigorous findings. According to Morse, this mixed approach helps “to obtain different but complementary data on the same topic” in order to best understand the research problem [27]. However, the study is not without limitations. One such limitation results from the use of thematic analysis of qualitative data. The flexibility of thematic analysis is known to lead to inconsistency and a lack of coherence when developing themes [47]. However, this was offset by being guided by methods and literature to coherently underpin the findings in this study. Again, in identifying the community participation, the study adopted retrospective approach which is based on community members' self-report. Given the time laps between implementation and study, the respondent could have forgotten some of the aspects of implementation. Similarly, respondent attitude during time of implementation could have been different from time of study.

## Figures and Tables

**Figure 1:** Level of community participation *N* = 400.

**Table 1:** Sociodemographic characteristics of community respondents (*N* = 400).

Variable	Frequency (*n*)	Percentages (%)
Age group		
15 to 24	46	11.5
25 to 54	277	69.3
55 to 64	39	9.8
Above 65	38	9.5
Gender		
Male	185	46.3
Female	215	53.8
Marital status		
Married	211	52.8
Unmarried	189	47.3
Education level		
No formal	41	10.3
Primary education	221	55.3
Secondary and above	138	34.5
Occupation		
Peasant	249	62.3
Formal employed	26	6.5
Others	125	31.3
Council		
Lindi MC	100	25
Nachingwea DC	100	25
Mtwara Mc	100	25
Nanyamba TC	100	25

**Table 2:** Community participation across demographic characteristics.

Variable	Community participation	
	Low *n*(%)	High *n*(%)
Age group		
15-24	38 (82.61)	8 (17.39)
25-54	240 (86.64)	37 (13.36)
55-64	30 (76.92)	9 (23.08)
65+	31 (81.58)	7 (18.42)
Gender		
Male	156 (84.42)	29 (14.6)
Female	183 (85.1)	32 (15.90)
Marital status		
Married	172 (81.52)	39 (18.48)
Unmarried	167 (88.36)	22 (11.64)
Education level		
No formal education	39 (95.12)	2 (4.88)
Primary education	180 (81.81)	40 (18.18)
Secondary and beyond	119 (87.0)	19 (13.0)
Occupation		
Peasant	212 (85.14)	36 (14.86)
Formal employed	21 (80.77)	5 (19.23)
Others	107 (84.80)	18 (14.20)
Councils		
Lindi MC	71 (71.0)	29 (29.0)
Nachingwea DC	83 (83.0)	17 (17.0)
Mtwara Mc	96 (96)	4 (4.0)
Nanyamba TC	89 (89)	11 (11.0)

**Table 3:** Distribution of score across each parameter.

Variable	No	Score	Yes	Score
Involvement in need assessment	349	0	51	51/400 = 0.1275
Organization	352	0	48	48/400 = 0.12
Volunteer for activity	387	0	13	13/400 = 0.0325
Program management	385	0	15	15/400 = 0.0375
Total/400	**—**	0	127/400	0.3175

Key: average score of 0 − 2 = low and 3 − 4 = high.

**Table 4:** Vector coordinators' viewpoint on community participation in biolarviciding (*N* = 12).

Variable	No *n* (%)	Yes *n* (%)
Involvement in need assessment	6 (50.00)	6 (50.00)
Organization	7 (58.33)	5 (41.67)
Resource mobilization		
Equipment	10 (83.33)	2 (16.67)
CORPS	10 (83.33)	2 (16.67)
Program management	11 (91.67)	1 (8.33)
Total/12	—	16/12 = 1.3

Key: average score of 0 − 2 = low and 3 − 4 = high.

**Table 5:** The level of willingness to participate in biolarviciding.

Variable	Frequency (*n*)	Percentages (%)
Likelihood to provide opinion		
Low	48	12.0
High	352	88.0
Likelihood to contribute fund		
Low	118	29.50
High	282	70.50
Contribution amount/year		
<5,000	329	82.25
5,000-10,000	17	4.25
11,000-15,000	1	0.25
>15,000	5	1.25
Likelihood to find time		
Low	96	24.0
High	304	76.0
Likelihood to participate in activities		
Low	66	16.50
High	334	83.50

**Table 6:** Logistic regression for predictors of community participation.

Variable	COR	95% confidence interval	*P* value	AOR	95% confidence interval	*P* value
Councils						
Lindi MC	Ref			Ref		
Nachingwea DC	0.50	0.26-0.99	0.046	0.417	0.20-0.87	0.002
Mtwara Mc	0.10	034-0.30	≤0.001	0.07	0.20-0.22	≤0.001
Nanyamba TC	0.24	0.11-0.54	0.001	0.22	0.09-0.52	0.001
Marital status						
Married	Ref			Ref		
Unmarried	0.569	0.072-0.644	0.054	0.35	0.18-0.69	0.02
Education level						
No formal education	Ref					
Primary education	9.111	1.217-8.210	0.997			
Secondary and beyond	6.387	0.828-9.241	0.998			
Occupation	Ref					
Peasant	1.409	0.499-3.975	0.517			
Formal employed	0.995	0.540-1.835	0.988			
Others						
Awareness	Ref			Ref		
No	2.47	1.33-4.58	0.004	1.68	0.78-3.62	0.185
Yes						
Willingness to participate	Ref			Ref		
Low	3.53	1.367-9.116	0.009	3.15	1.14-8.71	0.027
High						
Involvement	Ref			Ref		
No	5.128	2.668-9.856	≤0.001	6.07	2.69-13.71	≤0.001
Yes						

Note: Ref: reference category; COR: crude odd ratio; AOR: adjusted odd ratio.

## Data Availability

Data of this study can be obtained through sending request to massugii@gmail.com
